The article "Web Page Classification Algorithm Based on Deep Learning" was published in 2022. Journal: Comput Intell Neurosci.

# Web Page Classification Algorithm Based on Deep Learning

**DOI:** 10.1155/2022/9534918

**Published:** 2022-03-14

**Authors:** Yuanhui Yu

**Affiliations:** School of Computer Engineering, JiMei University, Xiamen 361021, Fujian, China

## Abstract

Transmit and process information to establish a learning mechanism and realize the processing of image data and sound data. However, the current research on Web page classification algorithm (WPCA) based on deep learning (DL) is not in-depth. Therefore, the main research of this article is the research of WPCA based on DL. This article first uses the keyword weight calculation method to reduce the impact of a small number of high-frequency words in the web page document on the weight calculation and reduces the value of the low-frequency word weights so that the WPCA is more accurate in the calculation process; second, the use of Chinese web pages: the classification method calculates the similarity between the text to be classified and all the class templates and then determines the category of all texts according to the similarity and certain classification rules; finally, in order to improve the learning rate of DL, consider using adaptive parameters. The optimization algorithm automatically adjusts the size of the learning rate, making the research of WPCA based on DL more efficient. After comparing the DL-based WPCA with the traditional algorithm, the data shows that in terms of time expenditure, the DL WPCA is 354 s, the traditional algorithm is 2436 s; in terms of memory overhead, the DL WPCA is 6.35 s, the traditional algorithm is 186.25 s. The experimental results show that WPCA based on DL are faster and more efficient than traditional algorithms and consume less system memory.

## 1. Introduction

### 1.1. Background and Significance

With the advent of the 5G era, the amount, dynamics, and complexity of online data continue to increase, and recommendation systems that can overcome the problem of excessive information begin to appear. At the same time, as DL has made gradual revolutionary advances in the fields of image analysis and speech recognition, it has also revolutionized industrial applications including recommendation systems. The deep learning algorithm is a network structure composed of multiple hidden layers. It mainly emphasizes the idea of “deep layer” and “layer-byftc-layer training.” After each layer is independently trained to obtain features, it continues to learn features as the input of higher layers. The process of extracting a high abstract representation: DL can directly extract functions from the content, process the data in the web page, has excellent phrase selection function, and can realize the modeling of dynamic data or sequence data. WPC is a process of determining the web page category of the tested web page by comparing the content and web page category of the tested web page according to the characteristics of the web page category. According to some mathematical algorithms, according to the user's use records, it is speculated that users can purchase items to achieve information search and filtering, which plays a particularly important role in today's dramatic increase in information.

WPC technology plays a very basic role in the download of web page information and belongs to the category of network content download. WPC research based on DL is crucial to applications such as directory website maintenance, topic browser construction, and search engine user experience improvement [1, 2]. One version that web users often appear in web page classifications is that portals generally display news at different locations on the homepage of technology and finance [3, 4]. Large-scale news makes manual classification unrealistic. At this time, accurate real-time news WPC technology will play a huge role [5]. Combined with the relevant technologies of current web page classification, referring to the establishment process of the text classification system, grab a certain amount of web page data and realize the automatic classification process for webpages. After the Chinese content is divided into words, each word is used as a feature. Through the appropriate feature weighting method, the vector space model is used to represent the feature vector of the web page, and the deep learning algorithm is used to train and model the web page training set for classification.

### 1.2. Related Work

Deep learning is a completely new field in machine learning research. Its essence is a multilayer perceptron with multiple hidden layers. It achieves extremely high accuracy through layer-by-layer initialization. It has been used many times in image recognition, speech recognition, text classification, and other fields. Shen et al. mainly research the latest advances in computer-aided image analysis and machine learning in the field of medical imaging, including deep learning to help identify, classify, and quantify patterns in medical images. The core of these advancements is the ability to use hierarchical functional representations learned only from data rather than manually designed features based on specific domain knowledge. DL is rapidly becoming the latest technology to improve the performance of various medical applications [6]. However, due to the limited literature he selected, the theory is not yet systematically matured. It is still in the preliminary research stage, and the experimental design is not yet complete. Oshea and Hoydis proposed and discussed several novel applications of DL in the physical layer. By interpreting the communication system as an autoencoder, a basic new method for treating the communication system design as an end-to-end reconstruction task was developed, aiming to unite the transmitter and receiver components in a single process. It showed how to extend this idea to a network composed of multiple transmitters and receivers and proposed the concept of a wireless transformer network as a means of integrating expert domain knowledge into a machine learning model [7].

### 1.3. Innovation in This Article

The main innovations of this paper include the following: (1) The new algorithm proposed in this paper can improve the accuracy and F1 value of web page classification and is an efficient WPCA. (2) Using the method of expanding web pages to add feature items and improve the accuracy of classification, this method is simple and easy to implement. The deep learning-based web page classification algorithm proposed in this paper may lose a low accuracy rate, but the classification efficiency is greatly improved, and the system overhead in the classification is also greatly reduced.

## 2. WPC Method Based on DL

### 2.1. Calculation of Keyword Rights for DL

After selecting functional items, it is necessary to weigh each item. As a result, the weight of more important clauses in the text will increase. There are many calculation methods for the weights of keywords, such as Boolean weights, weights based on the concept of the heir, weights of TFIDF type [8, 9], etc. The idea of the keyword extraction algorithm based on statistical features is to use the statistical information of the words in the document to extract the keywords of the document. Usually, the text is preprocessed to obtain a set of candidate words, and then keywords are obtained from the candidate set by means of feature value quantization. The most successful and widely used method in calculating the weight of keywords is “term frequency” (term “frequency” inverse document frequency), referred to as the tfidf method [10]. This method includes the importance of keywords in a document and the importance of the entire data set, combining the two into a single measurement.

It is usually calculated as follows:

(1) $$\begin{array}{c} i\;df_{k}=\log\left(\frac{N}{n_{k}}+0.01\right). \end{array}$$

Among them, *N* represents the total number of documents (text) in the data set: *n*_*k*_ represents the total number of documents containing the keyword *t*_*k*_. The weight *E* of a keyword *d*_*i*_ in document *w*_*ik*_ is calculated:

(2) $$\begin{array}{c} w_{tk}=tf_{i,k}*i\;df_{k}. \end{array}$$

Based on the if idf major, many scholars have proposed a “standardized” improvement method for this major. The improvement of tf is mainly to normalize the frequency of words and map them to the amount of interval [0,1] [11], which is as follows:

(3) $$\begin{array}{c} w_{ik}=\frac{{tf}_{i,k}*\;\log\left(\left(N/n_{k}\right)+0.01\right)}{\sqrt{\sum_{k=1}^{n}{\left(tf_{i,k}\right)}^{2}*\;\log^{2}\left(\left(N/n_{k}\right)+0.01\right)}}. \end{array}$$

The weight calculated by the above formula will often contain several items with larger values than other items. Because individual items with too high weights tend to hinder the influence of other items during the classification process, the frequency of statistical words needs to be properly balanced when calculating weights [12]. The weight calculation formula after word frequency equalization is as follows:

(4) $$\begin{array}{c} w_{i,k}=\frac{\sqrt{{tf}_{i,k}*\;\log\left(\left(N/n_{k}\right)+0.01\right)}}{\sum_{k=1}^{n}tf_{i,k}*\;\log\left(\left(N/n_{k}\right)+0.01\right)}. \end{array}$$

The formula of TF-IDF is only an empirical formula; there is no clear theoretical basis, and its physical meaning is not clear. TF-IDF is a statistical method to assess the importance of a word to a document set or one of the documents in a corpus. The importance of a word increases proportionally to the number of times it appears in the document but decreases inversely to the frequency it appears in the corpus. Various forms of TF-IDF weighting are often applied by search engines as a measure or rating of the degree of relevance between documents and user queries. Thorsten applied probability theory to TF-IDF, theoretically analyzed and explained, and obtained a new classification model. Shankar also improved TF-IDF [14]. Many people interpret TF-IDF from the perspective of word weighting and vector rotation and propose a method that uses an evaluation function to replace the weighted adjusted IN function in text feature selection [14]. Another commonly used normalization method, called the “log term frequency” method, uses the following formula to calculate the value of tf:

(5) $$\begin{array}{c} {tf}_{i,j}=\log\left({\text{freq}}_{i,j}\right)+1. \end{array}$$

The logarithmic word frequency method is the largest method of regularization coefficients for the frequency of text or word usage. The logarithmic function affects the word frequency through the value of tf, reducing the high frequency components of a few words in the document, reducing the impact on calculation, and the weight value of the frequency word, thereby reducing the influence of the change in document length on this value change [13, 15].

### 2.2. Chinese WPC Method

According to whether the learning is performed in the classification process, the automatic text classification technology can be divided into two categories of guided classification and unguided classification. The belt-oriented classification is also called domain classification or omission classification. It refers to the text categories determined in advance and provides text batches classified in advance for each text category, called the training set. In machine learning, samples are generally divided into three independent training sets: training set (train set), validation set (validation set), and test set (test set). Among them, the training set is used to build the model. The expression of the text class (i.e., class template) is determined according to the training set [13]. In actual classification, the similarity between the classified text and all class templates is calculated, and the type of all class texts is determined according to specific classification rules [16]. The type and number of texts are uncertain and can only be obtained after the compilation and aggregation of the texts. This classification method is called text clustering or undirected classification [17, 18]. Text aggregation usually adopts the hierarchical aggregation (system aggregation) method. This is often referred to as the coacervation method or bottom-up method. The outermost object of an aggregate is called the aggregate root, which is an entity. The aggregate root divides a clear boundary. Objects outside the aggregate root cannot directly access the internal objects of the aggregate root. If you need to access the internal objects, you must first access the aggregate root and then navigate to the internal objects of the aggregate. Initially, each text is considered a text category and then based on the text. In the same situation between those, the same text is often combined into one category. The other is called the decomposition method or the top-down method, which initially provides a rough classification of the entire text, and then becomes more concise. The text automatic classification technology described in this article refers to the classification with a guide. The following is the general process of automatic classification of Chinese text, as shown in Figure 1.

According to the general process of Chinese text classification shown in Figure 1, a classifier for classification can be constructed. The working principle of Chinese WPC is shown in Figure 2.

You can understand, according to Figure 2, the main work cycle of automatic text classification is divided into two stages of training and classification. During training, after the segmentation of Chinese words and feature selection processing, the examples of the training set will be expressed in the form of vectors come out. This feature vector group is used to describe the classification pattern in the classification process. After the Chinese web pages to be classified have undergone Chinese word segmentation and expressed as vectors, the classification algorithm is applied to the classification patterns obtained during the training process and a comparison is obtained. Next, the list of candidate categories is compared with the thresholds of each category obtained during the training process, and the categories larger than the threshold are stored and used as the classification result of the Web page.

### 2.3. Optimization Algorithm for Adaptive Parameters

The learning rate is a very important hyperparameter in DL and has a stupendous influence on the quality of the model. The learning rate is a hyperparameter that guides how we should adjust the weights of the network through the gradient of the loss function. The lower the learning rate, the slower the loss function changes. While using a low learning rate ensures that we do not miss any local minima, it also means that it will take us longer to converge, especially if we are stuck in a plateau region. Generally speaking, in DL applications, since the setting of the learning rate depends on artificial experience, it is often difficult for researchers to determine the reliable learning rate. Therefore, in order to automatically adjust the size of the learning rate, it is very meaningful to study the optimization algorithm of adaptive parameters. The most important function of the adaptive parameter optimization algorithm is that each parameter has a different learning rate and automatically adapts to these learning rates throughout the learning process. The AdaGrad algorithm is a general adaptive optimization algorithm. The global learning rate of the algorithm is *ε*, the initial parameter is *θ*, and the value *δ* (a small constant whose denominator is not zero) introduces a gradient cumulative quantity *r* (initialized to 0). In the training set, m samples {*x*_1_, *x*_2_, ..., *x*_*m*_} are randomly selected, the corresponding output is *y*_*i*_, the neural network mapping is represented as *f* (*x*; *θ*), and the loss function is *L* (*x*, *y*). Then the gradient calculation, gradient accumulation and parameter update are formulated as follows:

(6) $$\begin{array}{c} \hat{g}=\frac{1}{m}\nabla_{\theta }\sum_{i}L\left(f\left(x_{i};\theta \right),y_{i}\right),\\ r=r+\hat{g}\Theta \hat{g},\\ \theta =\theta -\frac{\varepsilon }{\delta +\sqrt{r}}\Theta \hat{g}. \end{array}$$

Among them, ⊙ is the Hadamard product of two vectors *A*(*a*_1_, *a*_2_,…,*a*_*n*_)^*T*^ and *B*(*b*_1_, *b*_2_,…,*b*_*n*_)^*T*^ with the same dimension, then *A*Θ*B*=(*a*_1_*b*_1_, *a*_2_*b*_2_,…,*a*_*n*_*b*_*n*_)^*T*^. Obviously, when the parameter has a large partial derivative, the learning rate will drop rapidly, and when the parameter has a small partial derivative, the learning rate drops slowly. However, in the process of increasing gradient accumulation, the learning rate will gradually approach zero, ending training early.

### 2.4. WPC Recommendation Model Based on DL

#### 2.4.1. Recommendation Model Based on Multilayer Perceptron

Multilayer Perceptron (MLP) is a simple but very effective feedforward neural network model. There are multiple hidden layers between the output layer and the intput layer. Widely used in the industrial field, it is also effective for recommender systems, as you can see, according to the three-layer MLP network structure in Figure 3.

#### 2.4.2. Recommended Model Based on Automatic Encoder

The autoencoder is composed of an input layer, a hidden layer, and an output layer. The number of neurons in the output layer is the same as the input layer, and the number of neurons in the hidden layer is less than the input layer. Such a structure allows the autoencoder to create a compressed representation of hidden layer data by learning data correlation. The data conversion from the input layer to the nondisplay layer is the encoding process *φ*, and the data conversion from the non-display layer to the output layer is the decoding process *φ*. The calculation method is shown in formulas (7) and (8).

(7) $$\begin{array}{c} \varphi :X⟶Z:x\mapsto \varphi \left(x\right)=\varphi \left(Wx+b\right)≔z, \end{array}$$

(8) $$\begin{array}{c} \phi :Z⟶X:\mapsto \phi \left(z\right)=\sigma \left(\tilde{W}z+\tilde{b}\right)≔x^{\prime }. \end{array}$$

Deep self-encoding is an enhanced version of a simple self-encoder with many hidden layers. The additional hidden layer allows the self-encoder to learn the deeper functions of the data. The first layer of the deep autoencoder can learn the first-level characteristical of the original input, and the second layer can learn the second-level characteristical corresponding to the first-level features. Applying deep self-encoding to more complex data, extracting feature information, performing score prediction and other activities, and combining with the recommendation system can obtain very good recommendation results.

#### 2.4.3. Model Based on Convolutional Neural Network

Convolutional neural networks (CNN) are good at processing topological data (such as grids) and can capture the global and local characteristics of the data. Almost all CNN-based recommendation systems use CNN to extract features. Weibo proposed an attention-based convolutional neural network model recommendation system for label recommendation. This is to consider the “#” tag as a multicategory classification problem. The model consists of global channels and local attention channels. The basic flow of the model is as follows: use convolutional layers and convolutional layers to obtain visual features from the image and inject user information to create personalized recommendations. You can use Bayesian personalized sorting algorithms to calculate the largest related labels.

#### 2.4.4. Recommendation Model Based on Recurrent Neural Network

Recurrent neural networks (RNN) are particularly suitable for recommendation problems, including evaluation and ranking related to recommendation systems. Recurrent Neural Networks can be trained using supervised and unsupervised learning theories. During supervised learning, the recurrent neural network uses the Backpropagation (BP) algorithm to update the weight parameters, and the calculation process can be analogous to the BP Through Time (BPTT) algorithm of the recurrent neural network. Recurrent neural networks for unsupervised learning are used for feature learning of structural information, and the most common form of organization is the Recursive Auto-Encoder (RAE). In many similar word reference systems or websites, it is difficult to obtain users' long-term consumption habits and long-term attention. At present, based on the interaction mechanism, the short-term preferences of users can be fully obtained, but this part of the data is very sparse and difficult to apply to the recommendation system. Recent progress shows that RNN is very efficient in solving this problem. Unlike feedforward neural networks, RNNs are calculated before loops and memories. Usually, barriers such as LSTM and GRU are actually used to overcome the problem of gradient disappearance.

#### 2.4.5. Recommendation Model Based on Deep Semantic Similarity Model

The Deep Semantic Similarity Model (DSSM) is inclusively used in the field of information search as a deep neural network, which is very suitable for the TOP-N recommendation. Given two sentences or text fragments, the task of text semantic similarity is to calculate the degree of semantic equivalence between them. As basic research in the field of natural language processing, text semantic similarity is becoming more and more important, and it is helpful for many applications in the field of natural language processing. In addition, text semantic similarity can also provide a unified framework for evaluating various other semantic components. The basic DSSM is composed of MLP, and more complex neural layers can be freely added if necessary, such as the convolutional layer and the largest wheeled layer. Project different items into a common low-dimensional space and use the cosine similarity calculation method to calculate the similarity of items.

#### 2.4.6. Emerging Methods: Neural Autoregressive Distribution Estimation and Generative Adversarial Networks

Neural autoregressive distribution estimation (NADE) estimates the true distribution of the source data and compares it with other DL-based recommendation models in some experimental data sets to obtain the best recommendation accuracy. Generative Adversarial Network (GAN) integrates the discriminant model and the generative model to maximize the advantages of both parties and generate better recommendation results.

## 3. Experiment of WPCSystem Based on DL

### 3.1. Experimental Environment

The experiment environment used in this article is as follows: the operating system is Windows10; the DL framework is TensorFlow-gpu, the version is v1.2.0; the IDE is Pycharm; the CUDA version is v8.0; the graphics card is NVIDIA GeForce GTX 1080Ti.

### 3.2. Experimental Procedure

This article proposes a new processing mechanism for web page information. The system has greatly improved the classification effect. This experiment will be divided into three parts to introduce compliance and design of the system. First, the processing flow of the WPC system is introduced, then the module design of the system is introduced, and finally, the test results of the system are discussed and analyzed.

1. The entire working cycle of the classifier can be divided into two parts: The training process and the classification process. In the training process, after the training set instance receives HTML tag analysis processing and the differentiation of Chinese words, the selection of feature items is expressed in vector form. This feature vector is used to illustrate the category pattern and is used in the classification process. The inspection set is part of the training set, and the interruption threshold for each category is determined in advance by applying the corresponding threshold strategy. During the classification process, the HTML files that are classified as Chinese web pages are analyzed and the Chinese word segmentation is processed. After being expressed as vectors, the classified algorithm obtains a comparative classification pattern during the training process to obtain a list of candidate categories. Compare the thresholds of each category and save the categories that are larger than the threshold to use as the classification result of the Web page. According to the characteristics of web page processing, the idea of module processing is proposed. The entire classification system is divided into four different modules: training document maintenance module, preprocessing module, feature extraction module, and feedback module.
2. Maintenance and management of educational document modules: Responsible for the management of educational documents for learning and extracting algorithms and functions. The main functions are creating and deleting document classes, adding, deleting, browsing, and indexing. The document set will be saved in a directory tree structure according to the category of the learning document.
3. Preprocessing module contains 2 submodules that can decompose HTML files and Chinese word segmentation. The HTML file phrase analysis submodule will remove invalid tags, attributes, and attribute values of HTML type web page conversion, text conversion, and HTML format functions. It will extract text information, location information, etc. The Chinese word segmentation simplified processing submodule uses a dictionary to decompose the educational document.
4. Feature extraction module: Feature item extraction refers to the selection of display terms and weight values in the target performance model. Use the dictionary to count the frequency of the words in the learning document, extract the function item set and related weight values of the document class according to the distribution of the word frequency, and generate a feature vector table.
5. Feedback module, that is, the threshold adjustment process. According to directory classification, domain name experts can correctly classify webpages classified in advance according to webpages or separators that have been classified in advance by inputting data, repeating tests, and adjusting critical values.

### 3.3. Training Data Set

In this paper, the 1200 pairs of depth-intensity map image pairs collected from the NYU-Depth V2 data set have too little data and the image resolution is too high to meet the training needs of the model. In order to increase the number of samples, this article first crops each pair of 640 × 480 resolution images to obtain 25 pairs of 128 × 128 resolution image pairs; and then rotates these 25 pairs of 128 × 128 resolution image pairs by 90 The operation of degrees, 180 degrees, and 270 degrees results in a total of 70,000 image pairs; finally, the 80,000 image pairs are mirrored to obtain the final 140,000 training samples.

## 4. Data Analysis of WPCA Based on DL

### 4.1. Analysis of WPC Effectiveness Based on Semantic Graph

This test is based on the DL and testing the effect of the WPC system. In the experiment, the entire contents of Table 1 and Figure 4 are used as a set of codes. The function word obtained through function selection is used as the function word set, and the text space after the word is used as the learning text space. Compared with the TF-IDF algorithm based on statistics, the WordRank algorithm based on the structured PageRank algorithm and view is finally used to train the classifier and form a classification pattern. Three indicators are used to test performance, namely: accuracy (*P*), recall speed (*R*), and F1. The test results are as follows.  Table 2 shows the *P* and *R* values of the three algorithms.  Figure 5 shows the performance test results of the F1 values of the three algorithms.

Comparing the *P* and *R* values of WPC according to Table 2 and comparing the F1 values of the weighting algorithms according to Figure 5, the following conclusions are drawn.

1. WPC comparison chart structure based on TF-IDF statistical algorithm PageRank-based WPCA has its own victory or defeat. In other words, for various types of web pages, some are in the category of statistics, and some are more sensitive to the meaning of words.
2. Compared with the TF-IDF and PageRank algorithms, the WordRank algorithm not only considers the statistics of word frequencies between web page categories but also considers the continuous morpheme coherence between texts. It combines two major categories of TF-IDF and PageRank algorithms. Advantages, thus showing excellent classification ability. In addition, the word vowel pattern is added to the text semantic logic chart. Because the phrase can display multiple words in the dictionary, the phrase range will become wider. Even if it is a word not included in the training bag, a word in this phrase will continue to be retained to provide classified information. It has great benefits for training with rich training content.
3. As can be seen from Figure 5, the WordRank algorithm has another advantage: relatively stable. Although functions are different, the algorithm can basically maintain a high level of algorithm, but the WPC, based on the TF-IDF algorithm, can basically reach 0.741, and the minimum value can reach 0.632, but the maximum sum of WPC based on the PageRank algorithm The minimum value can reach 0.632, the difference between the two is 0.286. Based on web page image design, using WordRank algorithm, based on statistical word frequency, combined with web page image analysis, can improve the stability of the algorithm.

### 4.2. Comparison of Data Classification Algorithms Based on DL and Traditional Methods

In order to verify the effectiveness of the DL-based WPCA proposed in this paper, this article will use DL-based WPCA and traditional classification algorithm to achieve WPC for comparison. It also compares the difference between the two classification algorithms in relation steps such as feature selection and vectorized representation of web pages.

1. In this experiment, the effect of the prior classification method on the classification algorithm will be tested, and a set of data will be tested within the range of the previously introduced data set, then 300 web pages will be randomly selected as the training set, and then the remaining part will be selected. Randomly select 150 web pages as the test set, as shown in Figure 6.
2. Through the comparison of experimental classification time, based on the consistency of the keywords proposed in this paper, you can see the method of WPC in advance, but it will not greatly improve the accuracy of web page classification, but also greatly improve the efficiency of web page classification. The comprehensive weighting calculation method previously proposed can be used for the selection of web page functions, which proves that it can effectively improve the accuracy ratio, recall speed and F1 value of web page classification. The selection of the DL function will display the function items that contain a lot of information and powerful recognition capabilities.
3. Based on previous experiments, the advanced method put forward in this paper tested the effect of the WPCA. The various optimization systems proposed in the test can effectively solve the shortcomings of the automatic classification algorithm applicable in the existing web page classification. This experiment will compare the classification quality and efficiency of the large-scale Chinese WPCA based on DL and the traditional WPCA and evaluate the classification algorithm proposed in this paper through the test results. The test conditions are shown in Table 3:

According to the above experimental data, when the nearest neighbor is set to 3, the hash code after the experiment is set to 48, and the size of the training set is 2000, the classification effect of these two classification algorithms is best. Using the above comparative test conditions, two different classification algorithms are used to classify 300 web pages, and the test results are shown in Figure 7.

After the above comparative tests, the influence of the web page preclassification method, CW-FS feature selection method, CW weight calculation method, and SH-FR method on the classification algorithm proposed in this paper were verified. The large-scale Chinese web page automatic classification algorithm based on DL is compared with the traditional web page automatic classification algorithm. Through the analysis of the experimental results, it can be shown that the DL-based web classification algorithm proposed in this paper may lose small accuracy, but the classification efficiency is greatly improved, and the system overhead in classification is greatly reduced. It is verified that the DL-based automatic WPCA proposed in this paper is more suitable for large-scale WPC than the traditional automatic WPCA.

## 5. Conclusions

The DL method proposed in this research can improve the efficiency of WPC and increase the stability of the WPCA. The second part of the experimental analysis is to compare the performance of the classification algorithm in different dimension feature spaces, compare the vector space, the efficiency, and time of the algorithm, for the purpose of proving the effectiveness of the function selection algorithm.

This paper proposes a method of expressing web page text as a weighted directed graph and constructing a semantic graph of the web page text. The establishment of the chart. Initially, the nodes of the characteristic language package chart are set as the bureau. Then, according to the construction requirements of similar edges and related edges, the words similarity and coword mining are used to describe the relevance between the words' information.

Aiming at the characteristics of the WPC structure under study, the contribution of the structural components is analyzed in detail according to the performance process of the web page. The feature extraction method of network files and the improved tf-idf algorithm based on web information fully illustrate the characteristics of the web page. This is used to represent a more typical vector space model of Web pages. Experiments demonstrate that the introduction of these methods can fully satisfy the actual demands of users [19].

## Figures and Tables

**Figure 1:** The general process of automatic classification of Chinese text.

**Figure 2:** Production principle of automatic classification of Chinese web pages.

**Figure 3:** Multilayer perceptron network structure.

**Figure 4:** Chinese web page classification data set.

**Figure 5:** FI value performance evaluation of WPC effect under three algorithms.

**Figure 6:** Impact of preclassification methods on classification algorithms.

**Figure 7:** Comparison test results.

**Table 1:** Chinese web page classification data set.

Serial number	Page genre	Number of training samples	Number of test samples
1	Game	521	236
2	Video	365	187
3	Newspapers	352	142
4	Transportation and Tourism	452	256
5	Medical health	476	219
6	Job search	325	203
7	Finance and Finance	403	174
8	Physical education	389	186
9	Educational culture	628	264
Total		3911	1867

**Table 2:** Estimation of *P* and *R* values of WPC effects under three algorithms.

Category	Evaluation index	TFIDF	PageRank	WordRank
Game	*P*	0.8147	0.7922	0.6948
	*R*	0.9058	0.9595	0.3171
Video	*P*	0.1270	0.6557	0.9502
	*R*	0.9134	0.0357	0.0344
Newspapers	*P*	0.6324	0.8491	0.4387
	*R*	0.0975	0.9340	0.3816
Transportation and Tourism	*P*	0.2785	0.6787	0.7655
	*R*	0.5469	0.7577	0.7952
Medical health	*P*	0.9575	0.7431	0.1869
	*R*	0.9649	0.3922	0.4898
Job search	*P*	0.1576	0.6555	0.4456
	*R*	0.9706	0.1712	0.6463
Finance and Finance	*P*	0.9572	0.7060	0.7094
	*R*	0.4854	0.0318	0.7547
Physical education	*P*	0.8003	0.2769	0.2760
	*R*	0.1419	0.0462	0.6797
Educational culture	*P*	0.4218	0.0971	0.6551
	*R*	0.9157	0.8235	0.1626

**Table 3:** Comparative test conditions.

	WPCA based on DL	Traditional WPCA
Feature selection	CW-FS feature selection method	Mutual Information MI Feature Selection Method
Feature weight	Comprehensive weight evaluation method	tf-idf weight calculation method
Dimensionality reduction method	SH-FR dimension reduction method	
Classification algorithm	KNN	KNN

## Data Availability

The data that support the findings of this study are available from the corresponding author upon reasonable request.
